The article "Application of a Depth Model of Precise Matching between People and Posts Based on Ability Perception" was published in 2022. Journal: Comput Intell Neurosci.

# Application of a Depth Model of Precise Matching between People and Posts Based on Ability Perception

**DOI:** 10.1155/2022/9040349

**Published:** 2022-09-22

**Authors:** Shaoze Zhang

**Affiliations:** ^1^Chinese Academy of Social Sciences, Beijing 100000, China; ^2^SEGi University, Kuala Lumpur, Malaysia

## Abstract

Under the modern environment, the reconstruction of enterprise's core competitiveness depends not only on capital and technical strength, but also on the overall strength of its human resources. At the same time, effective allocation and rational use of talents are needed to create good performance for enterprises. Enterprise human resource management is the key part of the whole enterprise management. At the same time, it is also a necessary preparation for the continuous development and innovation of enterprises. In the whole process of human resource management, the core work is person-post matching. Only by promoting the reasonable implementation of person-post matching can other management work be carried out smoothly. This paper expounds two major elements in human resource management, namely, the concept and measurement of person-post matching and the principle of person-post matching. And the factors in the matching of people and posts are analyzed. This paper probes into the implementation of person-post matching in enterprise human resource management. Based on this, this paper puts forward a depth model of accurate matching between people and posts based on ability perception. On the basis of studying the optimization of human resource scheduling, this paper takes into account three factors: resource constraints, heterogeneity of employee efficiency and time sequence relationship, and uses integer linear programming theory to model the system with the shortest construction period as the goal. The research shows that the accuracy of this algorithm can reach about 94%, which is about 8% higher than the traditional algorithm. It has certain superior performance. This will provide some reference for related researchers.

## 1. Introduction

With the advent of knowledge economy, human resources have become the most precious resources among all kinds of resources in enterprises. At the same time, the awareness of human resource management in enterprises has gradually improved. In the management of human resources, the matching of people and posts has gradually become a new topic in the development of enterprises [1]. The reconstruction of enterprise's core competitiveness depends not only on capital and technical strength, but also on the overall strength of its human resources. Facing the gradual formation of global economic integration, human resource management has become the core resource of enterprises. To ensure the sustainable development of enterprises, we must improve their core competitiveness through reform, attach importance to finding and solving many problems faced by human resource management, and promote the all-round development of enterprise reform [2]. It is not enough for an enterprise to accumulate human resources, but also to allocate and use them effectively in order to create good performance for the enterprise. At present, person-post matching usually refers to the matching degree between individual posts. It is both a verb and a noun, but it is regarded as a description of the allocation between individual employees and posts [3]. Generally speaking, the research on the structural dimension of person-post matching mainly considers five elements: employee ability matching, employee personality matching, job matching, job condition matching, and job reward matching. Under the trend of economic development, the positions of enterprises will also change with the changes of the market [4]. Different positions have different requirements for employees. The high matching between people and posts can improve the overall work efficiency of the enterprise, and the comprehensive level of the enterprise will be comprehensively improved, which is conducive to the long-term development of the enterprise.

The article "Application of a Depth Model of Precise Matching between People and Posts Based on Ability Perception" was published in 2022. Journal: Comput Intell Neurosci.

Person-post matching in human resource management of enterprises is to choose the right person to match the determined position, and at the same time take corresponding measures to combine the two. At the same time, it is necessary to adjust various problems in the process of combination, so as to ensure the realization of post objectives [5]. In the enterprise human resource management, the matching of people and posts plays an important role. In the process of enterprise development, the matching of people and posts can ensure the smooth implementation of enterprise strategic objectives. Every employee has subjective initiative, their work attitude determines the quality of work, and their willingness to work determines the work efficiency [6]. Even though the enterprise can provide employees with comfortable working environment, sufficient working resources and superior working conditions, if employees' willingness to work is low, the efforts made by the enterprise will be futile, and employees will still be unable to achieve higher working efficiency. Human resource management, for an enterprise in a fierce competition environment, is undoubtedly important. The human factor has been mentioned to a very important point in the enterprise, and the talents who manage the enterprise well have become a strategic behavior of enterprise development [7]. In the process of enterprise human resource management, post management is often influenced by many factors, including staff quality, enterprise planning, enterprise environment. And these factors are also controlled by the planning and design of jobs by enterprises, so as to better realize the complete match between individuals and jobs [8]. Person-post matching in human resource management can not only ensure the normal operation of enterprises, but also comprehensively improve the comprehensive quality of employees, which is also an important advantage for improving the competitiveness of enterprises.

The article "Application of a Depth Model of Precise Matching between People and Posts Based on Ability Perception" was published in 2022. Journal: Comput Intell Neurosci.

Higher work efficiency is the result of the joint efforts of employees and organizations. However, in the process of improving employees' job performance, many enterprises often only consider organizational factors, while ignoring employees' personal factors. In fact, personal factors may have more influence on job performance than organizational factors. Through effective person-post matching, the quality of enterprise resource management can be comprehensively improved, which plays an important role in enterprise operation and work development. It is also very helpful for enterprises to achieve strategic goals [9]. In fact, the matching between people and posts usually needs to effectively integrate the personal characteristics of employees with the overall characteristics of posts, so as to achieve the most ideal human resource management effect. Based on the current situation of human resources management in enterprises, this paper mainly focuses on optimizing the allocation of personnel and posts in enterprises, realizing the precise matching of personnel and posts, and giving full play to the effective allocation of human resources management, so as to effectively improve work efficiency. In this paper, a depth model of accurate matching between people and posts based on ability perception is proposed. On the basis of studying the optimization of human resource scheduling, this paper takes into account three factors: resource constraints, heterogeneity of employee efficiency and time sequence relationship, and uses integer linear programming theory to model the system with the shortest construction period as the goal. Aiming at the shortcomings of the algorithm, an improved genetic algorithm is proposed. The research shows that the crossover strategy of priority set is adopted in the crossover process of the improved genetic algorithm, and the algorithm can be solved quickly.

Based on ability perception, this paper analyzes the application of person-post precise matching depth model. This paper expounds the two elements of human resource management, namely, the concept of person-post matching, measurement and the principle of person-post matching, and analyzes the factors that affect the person-post matching. The research is divided into five parts. The first part expounds the post responsibilities and the development background of the post. The second part expounds the post' economic benefits of the enterprise. It provides some references for relevant researchers. The third part analyzes the person-post matching in human resource management. The fourth part discusses the result analysis. The person-post exact matching model studied in this paper can not only improve the work efficiency of employees, but can also promote the development of enterprises and bring considerable economic benefits to enterprises.

The article "Application of a Depth Model of Precise Matching between People and Posts Based on Ability Perception" was published in 2022. Journal: Comput Intell Neurosci.

## 2. Related Work

In today's situation of global economic integration, if we want to survive and develop, we must attach importance to human factors. Therefore, we should pay attention to strengthening the management of human resources in enterprises. At present, many scholars have discussed the related content of human resource management.

Grigorescu et al. believe that in order to realize the matching of people and positions, first of all, it is necessary to have a thorough understanding of the talents and interests of employees, so as to select suitable candidates for a specific position and let the right people do the right things, only in this way can people achieve the effect of post matching [10]. Popaitoon and Siengthai proposed a dynamic human resource management model. It believes that human resource management should be based on mature and perfect management factors according to the development characteristics of different industries, according to the company's own situation and its specific organizational form and work nature, in the dynamic changing market environment, the organization design, human resource management of job analysis, job setting, performance evaluation, selection configuration, and incentive mechanism [11]. Taking scientific research and design units as the research object, Pelit and Katircioglu constructed a model of the relationship between person-post matching, insider identity perception, innovation self-efficacy, and employee innovation behavior and demonstrated the model through multiple linear regression. The research results show that Person-post matching positively affects employees' innovative self-efficacy and innovative behavior [12]. Combined with the four-dimensional structural model of job performance, Graham et al. refined the job performance into two dimensions, namely, task performance and learning performance, and comprehensively considered employees' existing performance and future development potential [13]. Fox and Cowan proposed to combine the scientific concept of development, establish a people-oriented human resource management concept, adhere to the coordinated development of individuals and society, and realize the innovation of human resource management. The development and management of the system are truly scientific [14]. This paper matches the post's analysis and personnel on the basis of scientific analysis, and organically combines human resource management systems and systems, such as performance management system, post evaluation system, salary system, career management and promotion system, training and development system, and competitive employment system. Compared with the traditional personnel management institute, it provides more favorable support for the realization of the overall strategic objectives of the unit. Starting from the operability, based on the method of systematic analysis and quantitative evaluation, Aino et al. established an optimal allocation model of human resources. It provides a specific method of quantitative management for the optimal allocation of human resources [15]. From the institutional perspective of the theory of public service motivation, Tung proved that person-post matching can improve public service motivation, and public service motivation is between the positive effect of person-post matching on employee satisfaction [16]. Geneviève et al. designed the scales of person-post fit, perceived obligation, and job performance based on a large number of references and research purposes, as well as the nature of the companies studied [17]. Wu et al. believe that person-post matching can improve employee organizational commitment, organizational citizenship behavior and job satisfaction, and can reduce employee turnover willingness [18]. Esat et al. used perceived obligation as a moderator variable to study the relationship between person-post fit and job performance [19]. Peng and Mao conducted a survey on a company's leaders and their employees, and used a hierarchical linear regression model to analyze that there is a significant positive correlation between person-post matching and employee task performance [20]. Cyclic neural network is a kind of artificial neural network, which can create cycles in the network graph by adding additional weights to the network in order to maintain an internal state. The advantage of adding states to neural networks is that they will be able to clearly learn and use context in sequence prediction problems, including problems with sequence or time components.

The article "Application of a Depth Model of Precise Matching between People and Posts Based on Ability Perception" was published in 2022. Journal: Comput Intell Neurosci.

Based on the in-depth study of related literature, this paper constructs a depth model of precise matching between people and posts based on ability perception, starting from the relationship among people and posts matching, perceived obligation and job performance. And on the basis of building a relatively perfect system of personnel and posts, using natural language processing technology and Doc2vec method, we can fully mine the semantic information contained in long texts, and realize the accurate matching of information between talents and posts. At the same time, in order to solve the problem of unreasonable allocation of multi-skilled personnel, a resource allocation strategy based on the maximum overlapping task set is proposed to allocate human resources. The research shows that the algorithm in this paper can be solved quickly, which is beneficial to realize more accurate and personalized accurate matching of people and posts.

## 3. Methodology

### 3.1. The Matching of People and Posts in Human Resources Management

In the process of enterprise development, personnel competition is inevitable. In the process of human resource management, healthy competition can not only strengthen the management of matching people with posts, but also promote the development of enterprises. To achieve this, in the process of human resource management, the principle of fairness must be followed in the matching of people and posts [21]. In addition, we should follow the principle of balance between people and posts. Person-post balance not only refers to the correspondence between employees and posts in quantity, but also refers to the correspondence between post level and employee's ability level. In the actual optimal allocation of human resources, it is necessary to select and allocate them according to the specific situation of the organizational structure and the emphasis of the position on the ability requirements of staff. Usually, it is necessary to consider the candidates' scores on various competency elements required by their positions, and the weight distribution of each competency element in different positions. Job analysis is also called job analysis. It refers to a complete description or description of a work in order to provide information about positions for human resource management so as to carry out a series of basic activities of post information collection, analysis, and comprehensive human resource management. Many enterprises have paid a great price for the lack of accurate job descriptions, resulting in a lot of human resources work.

By analyzing the job content of a post, it is convenient for human resource managers to understand the environment, tasks, and responsibilities of the post, so that they can make effective matching when the posts are distributed. Competence refers to the knowledge, skills, and experience of employees engaged in a specific job. It is a relatively stable personal trait that determines their job performance. Employees' abilities mainly include their ability to complete work and solve problems, etc. Enterprises should strengthen staff training and improve their professional skills. In terms of training methods, we should combine theory with practice, not only focus on improving employees' knowledge level, but also enrich employees' actual combat experience. In terms of training content, targeted training should be provided to employees according to job requirements and job nature. The accurate matching algorithm of people and posts based on ability perception is shown in Figure 1.

The article "Application of a Depth Model of Precise Matching between People and Posts Based on Ability Perception" was published in 2022. Journal: Comput Intell Neurosci.

In the process of enterprise development, it is imperative to divide the human resources in order to realize the matching of people and posts. In a specific period, the demand for employees and related forecasts needs to be planned according to the actual situation of enterprise development. The concept of competency includes three meanings: deep-seated characteristics, causality, and criterion reference. A complete post competency evaluation system should not only be relatively scientific and reasonable in theory, but also be operable. Therefore, after establishing the post competency model and selecting the evaluation tools, we will enter the implementation stage of post competency evaluation. At the same time, enterprises should strengthen the management of human resources, rationally allocate employees according to the job requirements, and ensure that the quantity and quality of employees match the job requirements. Talent evaluation is the basis of job matching. In the process of human resource management, enterprise managers should evaluate candidates in all aspects, and make job matching according to their abilities. When an enterprise selects employees for a position, it needs to know the duties and qualifications of the position. The job analysis analyzes the position from the perspective of responsibility and authority, and then describes the analyzed position in the form of job description, as well as the requirements of the position on knowledge, skills, and abilities.

Individuals with a high degree of job matching believe that their innovative ability can meet job requirements and that they can successfully adopt innovative ideas and ideas to solve problems at work, that is, they have a high sense of innovative self-efficacy. On the contrary, employees with low job-to-job matching show low self-confidence in work innovation because their innovative ability cannot meet the needs of their jobs, that is to say, their innovative self-efficacy is low. In addition, in the enterprise operation, the working hours and working ability of employees will change. In the process of work, if the employees of the enterprise perform well and the performance of the assessment is outstanding, the enterprise should adjust the positions of employees according to its own development. Make new employment opportunities and manage new positions effectively, which can promote the development of enterprises. At the same time, we should improve the internal promotion channels and fully care about the personal development of employees. On the one hand, it is necessary to strengthen the vocational training of employees, improve their personal abilities and help them achieve personal promotion. On the other hand, help employees to make their own career plans according to the company's career path, encourage employees to learn from their strengths and avoid their weaknesses, and point out their career development direction for employees.

The article "Application of a Depth Model of Precise Matching between People and Posts Based on Ability Perception" was published in 2022. Journal: Comput Intell Neurosci.

### 3.2. Construction of Depth Model of Accurate Matching between People and Posts Based on Ability Perception

In this chapter, the depth model of accurate matching between people and posts based on ability perception is constructed. There are two meanings in the accurate matching of posts: first, posts must have their talents, that is, the abilities required by posts need to be fully possessed by someone. Second, people need their posts, that is, employees have the ability to be fully qualified for this post. In the filtering layer of quantitative calculation, this paper first quantifies the related features of the posts, and then uses the numerical comparison calculation method to determine the matching degree of the related features. Because different positions have different responsibilities and different requirements for personnel's ability, it is necessary to determine the weight distribution of various ability elements in each position. The method of Doc2vec is used to vectorize the attribute values with long text in the matching features of people and posts, and then the matching degree of the corresponding features is evaluated by calculating the cosine distance between the corresponding features. In this paper, some infeasible solutions are allowed to exist and others are heuristically modified, that is, on the one hand, the infeasible solutions are tolerated in the population through penalty function mechanism, and on the other hand, some infeasible solutions are selected to be modified. Weighting in the behavioral feature layer, through job seekers' operations, such as post delivery and collection, weighting processing is carried out on the previous pure post-feature attributes. In the research of related algorithms for solving multi-skilled human resource scheduling problems, there are mainly mathematical programming and intelligent optimization algorithms. Mathematics is generally used to solve small-scale optimization problems. As the scale of the problem increases, it is often impossible to find the optimal solution in a reasonable time. Intelligent optimization algorithm has the characteristics of simple description, strong robustness and easy implementation. The scheduling process of multi-skilled human resources in this paper is shown in Figure 2.

The article "Application of a Depth Model of Precise Matching between People and Posts Based on Ability Perception" was published in 2022. Journal: Comput Intell Neurosci.

The foundation of person-post matching model lies in the establishment of person-post characteristic system. Job characteristics system is mainly constructed according to the information needs of both job seekers and enterprises. According to the information needs of job seekers and enterprises, the characteristics of enterprise posts and job seekers can be constructed. In order to ensure the scientificity and fairness of the evaluation, we should generally consider various evaluation factors and their respective weights in the evaluation, because the sample size of modeling data is generally large. But in practice, including too many variables will also have some side effects. If too many items are set in the post application form or leader evaluation form, the accuracy of the answer will be reduced. A common way to overcome this problem is to examine a large number of variables first, and then select them. For multi-objective function processing, there are generally two methods in genetic algorithm. First, several objective functions are integrated into a new objective function by weighting. The second is to satisfy multiple objective functions through priority order. In this paper, the method of comparing multi-objective functions in priority order and arranging individual order is adopted, which has strong practical application value. Job characteristics refer to the construction of job characteristics, mainly including job situation and job requirements, and most of its attributes can reflect the characteristics and needs of this job. Job seekers' characteristics mainly include job requirements, while enterprises pay attention to job seekers' basic information, job-seeking intention, educational background, mastery of skills, work experience and personal evaluation. Its characteristic attributes reflect the background information and job-seeking willingness of job seekers themselves. A multi-objective optimization problem can be expressed as follows:

(1) $$\begin{array}{c} \text{min}F\left(x\right)=\left(f_{1}\left(x\right),f_{2}\left(x\right),f_{3}\left(x\right),\ldots ,f_{k}\left(x\right)\right), \end{array}$$

(2) $$\begin{array}{c} s.t.g_{i}\left(x\right)\leq 0,1,2,3,\ldots ,m,x\in \Omega . \end{array}$$

Among them, *x* is the *n* -dimensional decision vector (*x*=*x*_1_, *x*_2_, *x*_3_,…, *x*_*n*_, ); the target vector *F*(*x*) contains *k* targets *f*_*i*_(*x*); *g*_*i*_(*x*) is the constraint condition; *Ω* is the feasible region.

The article "Application of a Depth Model of Precise Matching between People and Posts Based on Ability Perception" was published in 2022. Journal: Comput Intell Neurosci.

This algorithm is based on the penalty function, and uses the probability *P*_*f*_ to correct some non-feasible solution individuals. The penalty function integrates the three constraints with the objective function to form a new objective function:

(3) $$\begin{array}{c} \begin{array}{c} J_{1}^{\prime }\left(X\right)=J_{1}\left(X\right)+\overset{2}{\underset{t=1}{\sum }}\lambda_{i}{\left[D_{i}\left(t\right)-X_{i}\left(t\right)-\pi_{3i}X_{3i}\left(t\right)\right]}^{+}\\ +\lambda_{3}{\left[D_{3}\left(t\right)-X_{3}\left(t\right)+X_{31}\left(t\right)+X_{32}\left(t\right)\right]}^{+}\\ +\lambda_{4}{\left[X_{3}\left(t\right)-{\tilde{X}}_{M}\right]}^{+}. \end{array} \end{array}$$

Among them, *λ*_1_, *λ*_2_, *λ*_3_, *λ*_4_ are penalty function factors, which can be adjusted according to the actual situation. After training, obtain document vectors of feature attributes corresponding to job applicants or positions. Then, the similarity of corresponding feature attributes is obtained by calculating the cosine distance between documents. Finally, the matching degree of text similarity computing layer features is obtained by accumulating. The formula is as follows:

(4) $$\begin{array}{c} S_{i⊗j}=\frac{V_{i}\times V_{j}}{\left\|V_{i}\right\|\times \left\|V_{j}\right\|}, \end{array}$$

(5) $$\begin{array}{c} p_{doc}=S_{i1⊗j1}+S_{i2⊗j2}+S_{i3⊗j3}. \end{array}$$

Among them, *V*_*i*_ represents the document vector of the feature attribute *i*, *V*_*j*_ represents the document vector of the feature attribute *j*; *S*_*i*1⊗*j*1_ represents the similarity of the feature attributes *i* and *j* long texts; *p*_*doc*_ represents the similarity of the text similarity calculation layer between the job seeker and the post.

Let *R*_*m*_ be the *m*th employee with heterogeneous skills and efficiency; *C*_max_ is the shortest project duration; *p*_*jv*_ is the time required by the employee *v* to process the task *j*; *UB* is the longest time for the employee to complete all tasks. But:

(6) $$\begin{array}{c} MinC_{\text{max}}=\left\{FT_{j}|j\in J\right\}. \end{array}$$

Equation (7) satisfies the completion time of each task. The completion time should be no less than its actual processing time.

(7) $$\begin{array}{c} FT_{j}\geq \overset{UB}{\underset{r=1}{\sum }}p_{jv}x_{jvr},\forall j\in J,\forall v\in M. \end{array}$$

The decision variables are:

(8) $$\begin{array}{c} x_{jvr}=\left\{\begin{array}{c} 1,\forall j\in J,\forall v\in M,\forall r\in R,\\ 0. \end{array}\right. \end{array}$$

There are also feature attributes described by long texts in the characteristics of posts, and these corresponding long texts describe the specific ability requirements of posts and the skills of job seekers, which are the key information for accurate matching between posts and job seekers. The deep semantic information implied in the long text reflects the characteristics of job seekers or posts. The purpose of introducing penalty function in this paper is to reduce excessive human intervention in genetic operation in order to find feasible solutions, and to reduce the probability of infeasible solutions being selected for genetic operation in the population, but it is impossible to fundamentally avoid the existence of infeasible solutions.

The article "Application of a Depth Model of Precise Matching between People and Posts Based on Ability Perception" was published in 2022. Journal: Comput Intell Neurosci.

## 4. Result Analysis and Discussion

In the process of enterprise development, human resource management is very important. Employees are the foundation of an enterprise's production and operation. In this process, the matching between people and posts plays a key role. Based on the perspective of human resource management, the last section constructs a depth model of precise matching between people and posts based on ability perception. In order to verify the performance of the model, experiments are carried out in this paper. First, set the initial value of dynamic adaptive change to 0.1, the change rate to 1.06 and the threshold to 0.2. In the experiment, three performance evaluation indexes are adopted, namely, average absolute error, recall rate, and F1 value. They are two metrics widely used in the field of model performance testing to evaluate the quality of results. Through experiments, the results of each index of this model are obtained, and then compared with other models to verify the reliability and superiority of this method. Comparison of average absolute errors of different models is shown in Figure 3. Comparison of recall rates of different models is shown in Figure 4. Comparison of F1 values of different models is shown in Figure 5.

It can be seen that the average absolute error of this model is low. The recall rate and F1 value are high. This result verifies the reliability and superiority of this method. In this paper, on the basis of qualitative analysis of personnel and positions, combined with quantitative analysis, the optimal allocation scheme is selected. It can better optimize the personnel structure of the organization and improve the overall efficiency of the organization. The mean, standard deviation, and correlation coefficient of each variable in this paper are given in Table 1.

The article "Application of a Depth Model of Precise Matching between People and Posts Based on Ability Perception" was published in 2022. Journal: Comput Intell Neurosci.

It can be seen from the table that the generalized distance value obtained by this algorithm is smaller than the other two algorithms, which indicates that the performance of this algorithm is better than that of MOCS algorithm and IMOCS algorithm. The key point of genetic algorithm in solving scheduling problem lies in the solution representation method, that is, designing the solution structure. In this paper, decimal coding is adopted, and the objective function of shortest duration is selected as the fitness value function of genetic algorithm. The advantage of this is that it is very intuitive, and excellent individuals have the shortest construction period. The accuracy of human resource scheduling with different algorithms is shown in Figure 6.

The results show that the performance of this algorithm is better. This method provides a strong theoretical basis and reference for human resource scheduling, and has practical significance. In order to verify the effectiveness of this algorithm again, the performance of this algorithm is compared with that of MOCS algorithm and IMOCS algorithm. In order to ensure the rigor and reliability of this research, this paper calculates the generalized distance values of different algorithms under the same conditions.  Table 2 shows the generalized distance values obtained by different algorithms.

Incorporate the evaluation results into the further career development of employees. This method can promote the learning enthusiasm of internal employees and provide good help for their career planning. At the same time, enterprises can quantitatively assess employees, so that capable employees can work in more challenging positions. Through module analysis, the following results can be obtained:

1. If the qualification of the employee is completely consistent with the requirements of the post, it meets the requirements of the post,
2. If the qualification of the employee does not meet the post requirements (for example, the employee's understanding of the financial product is lower than the post needs of the customer manager). At this time, you can prompt the employee to carry out relevant training. And provide the corresponding system link, for example, the employee does not have project management related skills, which does not meet the requirements of the post.
3. The qualification of staff's proficiency is higher than the post needs, for example, the staff's understanding of the financial product is higher than the post needs of the customer manager.

The article "Application of a Depth Model of Precise Matching between People and Posts Based on Ability Perception" was published in 2022. Journal: Comput Intell Neurosci.

Person-post matching has a significant positive effect on job performance. Without considering other factors, improving person-post matching can improve employees' job performance. Perceived obligation has a significant positive moderating effect on the relationship between job matching and job performance, that is to say, the stronger perceived obligation is, the better job performance can be achieved by improving job matching. In this paper, we test the matching accuracy of person-post precision matching model, and the results are shown in Figure 7.

The results of this paper are the same as those actually obtained. This shows that this algorithm can get the optimal solution of the problem quickly, has obvious advantages when there are many people and posts, improves the efficiency of personnel allocation, and is an effective algorithm to solve the problem of optimal allocation of human resources.

## 5. Conclusions

With the continuous development of economy and the expansion of economic market, if an enterprise wants to become bigger and stronger, it must first have a clear understanding of employees' professional skills and interests. Only in this way can the matching between employees and posts be truly achieved. At the same time, with the shift of strategic objectives of enterprises, job responsibilities and job requirements will also change, and people's quality and ability are constantly changing. Therefore, the matching between people and posts is dynamic. On the basis of studying the optimization of human resource scheduling, this paper takes into account three factors: resource limitation, heterogeneous employee efficiency and time sequence relationship, and uses integer linear programming theory to model the system with the shortest construction period as the goal. In this way, accurate matching of personnel and posts and scheduling optimization can be realized. The research shows that the accuracy of this algorithm can reach about 94%, which is about 8% higher than the traditional algorithm. It has certain superior performance. The precise matching model of people and posts studied in this paper can not only improve the work efficiency of employees, but also promote the development of enterprises and bring substantial economic benefits to enterprises. This will provide some reference for related researchers. In addition, the accurate matching of people and posts is a relatively complicated process. To do this, enterprises need to optimize the distribution of posts in the process of development, combining with their own development, so as to improve the matching degree of people and posts. This will help enterprises reduce the cost of employing people, fully mobilize the enthusiasm of employees, accelerate the development rate of enterprises and realize the rapid progress of the economic market. This paper also needs to analyze the existing human resource information system. At present, there are some deficiencies in the person-post matching module in the human resource information system. There is no idea to build the person-post matching scoring model according to the abilities of different employees. In the future, specific analysis and design are needed for this point. [22].

The article "Application of a Depth Model of Precise Matching between People and Posts Based on Ability Perception" was published in 2022. Journal: Comput Intell Neurosci.

## Figures and Tables

**Figure 1:** Accurate matching algorithm of people and posts based on ability perception.

**Figure 2:** Flow chart of multi-skilled human resource scheduling.

**Figure 3:** Comparison of average absolute errors of different models.

**Figure 4:** Comparison of recall rates of different models.

**Figure 5:** Comparison of F1 values of different models.

**Figure 6:** Accuracy of different scheduling algorithms.

**Figure 7:** Matching accuracy results of person-post.

**Table 1:** Mean value, standard deviation, and correlation coefficient among variables.

Variable	M	SD	1	2	3	4	5	6
Gender	1.45	0.489						
Age	1.98	0.697	0.09					
Degree of education	2.60	0.754	−0.061	−0.018				
Length of service	2.75	1.513	−0.023	0.623^*∗∗∗*^	−0.361^*∗∗*^			
Position rank	1.84	0.894	−0.019	0.221^*∗∗*^	0.079	0.451		
Person-post matching degree	3.59	0.841	−0.039	0.237^*∗∗*^	−0.068	0.282^*∗∗∗*^	0.179	
Ability perception	3.52	0.885	0.134	0.189^*∗∗*^	0.083	0.109^*∗∗*^	0.187^*∗∗*^	0.301^*∗∗*^

**Table 2:** Generalized distance values of different algorithms.

Algorithm	SCH	ZDT1	ZDT2	ZDT3	LZ
MOCS algorithm	1.27E-07	1.21E-07	2.31E-05	2.87E-05	4.26E-05
IMOCS algorithm	1.29E-07	1.08E-07	1.58E-07	2.94E-05	3.28E-05
Algorithm in this paper	7.34E-09	1.06E-07	1.43E-07	3.18E-07	3.16E-05

## Data Availability

The data used to support the findings of this study are available from the corresponding author upon request.
